# Treatment of chronic hepatitis C with sofosbuvir in a hemodialysis patient: a case report

**DOI:** 10.11604/pamj.2021.38.137.20560

**Published:** 2021-02-08

**Authors:** Marius Djoumbissie Tchoupe, Hanen Chaker, Mona Boudabbous, Salma Toumi, François Pegdebamba Kissou, Saba Gargouri, Khawla Kammoun, Faiçal Jarraya, Nabil Tahri, Soumaya Yaich, Mohamed Ben Hmida

**Affiliations:** 1 Nephrology Department, Faculty of Medicine, Hedi Chaker University Hospital and UR 12ES14, Sfax, Tunisia,; 2 Hepato-Gastroenterology Department, Hedi Chaker University Hospital, Sfax, Tunisia,; 3 Microbiology Laboratory, Habib Bourguiba University Hospital, Sfax, Tunisia

**Keywords:** Hemodialysis, hepatitis C, treatment, sofosbuvir, case report

## Abstract

The treatment of chronic hepatitis C virus (HCV) infection in chronic hemodialysis patients remains an issue of great concern for nephrologists. In 2008 the kidney disease improving global outcomes working group suggested the use of pegylated interferon in end stage kidney disease patients treated by dialysis. Since then, series and some clinical trials on different direct-acting antiviral agents have shown better efficacy and tolerance than interferon-based regimens. Data on the efficacy, tolerance and the right dose of sofosbuvir in this population are still unclear. We report a case of chronic HCV genotype 1b infection in a 47-year-old patient on maintenance hemodialysis successfully treated by a combination of sofosbuvir and ledipasvir for 12 weeks. Evolution was marked by the complete regression of the hepatic cytolysis, a complete and sustained virologic response with HCV viral load undetectable for a 24 months follow-up period. No adverse reaction was found. The treatment of HCV genotype 1 or 4 infection in patients on maintenance hemodialysis is possible with sofosbuvir based regimens with a good efficacy/safety ratio in the absence of current recommended drugs for patients with eGFR<30ml/min/1.73m^2^. The prescription of sofosbuvir should be encouraged amongst this population in this setting.

## Introduction

Hepatitis C virus (HCV) infection is much more prevalent in patients on renal replacement therapy than in the general population [1]. Indeed, it is associated with an increased risk of mortality in these patients [2]. In 2008, the kidney disease improving global outcomes (KDIGO) working group suggested the use of pegylated interferon in end stage renal disease (ESRD) patients treated by dialysis [1]. However, treatment outcomes were poor and side effects sometimes intolerable. Since then, case series and some clinical trials on different direct acting antiviral agents (DAAs) have shown better efficacy and tolerance than interferon based regimens. Sofosbuvir is not recommended for use in patients with estimated glomerular filtration rate (eGFR) <30 ml/min/1.73 m^2^ [3,4]. More data are needed to expand the prescription to this population [3]. Data are accumulating on the use of sofosbuvir (SOF) in patients with low eGFR and particularly in patients on maintenance hemodialysis (HD). Nevertheless, data on the efficacy, tolerance and the right dose of sofosbuvir in this population are still unclear. We report a case of chronic HCV genotype 1b infection in a patient on maintenance HD successfully treated by a full dose combination of sofosbuvir and ledipasvir at Hedi Chaker University Hospital, Sfax, Tunisia, the only DAAs combination currently available.

## Patient and observation

A 47-year-old patient has been undergoing maintenance HD for 32 years. The underline nephropathy was an undetermined chronic glomerular disease. He was anuric with no renal transplantation plan. There was a history of multiple blood transfusions during the first 5 years of HD and no scarification. Complications of ESRD included secondary hyperparathyroidism with parathyroidectomy in 2012 for refractory secondary hyperparathyroidism to medical treatment. Long-term complication of HD was beta 2 microglobulin amyloidosis with shoulder destructive arthropathy and bilateral carpal tunnel syndrome. He was tested negative for HIV and he had a naturally acquired hepatitis B immunity. Moreover, a chronic HCV genotype 1b infection was diagnosed at the 25^th^ year of HD treatment and there was no tendency for spontaneous resolution: positive HCV serology, positive HCV polymerase chain reaction, gradual increase of viral loads from 6.17x10^5^ to 1.5x10^7^ IU/ml (Table 1) and hepatic cytolysis (1.5 to 2 upper limit of normal). There were no signs of hepatocellular insufficiency or portal hypertension. The Liver remained homogenous with normal size and there was no extrahepatic HCV infection related manifestations. After a multidisciplinary approach and the written consent of the patient, a specific antiviral treatment with a Sofosbuvir based regimen was started. It featured: sofosbuvir and ledipasvir 400/90mg: 1 tablet daily for 3 months, the only DAAs combination currently available. Evolution was marked by the complete regression of the hepatic cytolysis syndrome, a complete and sustained virological response (SVR) with HCV viral load undetectable from the 12^th^ week of treatment to the time of this report (24 months later). No adverse reactions were reported.

**Table 1:** liver function tests and virological profile

	Before treatment					During treatment	After treatment
	2011	2013	2014	2015	2016	2017 (12^th^ week of treatment)	2019
HCV viral load (x10^6^IU/ml)	0.617	-	4.95	14.80	15.00	UD	UD
Serum ASAT (IU/l)	-	23	20	21	62	10	14
Serum ALAT (IU/l)	-	25	19	23	27	7	3
Serum ALP (IU/l)	-	74	91	80	79	64	72
Total serum bilirubin (mg/l)	-	5	4	6	6	9	11
Serum gamma GT (IU/l)	-	23	22	23	18	15	14

HCV: hepatitis C virus; ASAT: aspartate aminotransferase; ALAT: alanine aminotransferase; ALP: alkaline phosphatase; GT: glutamyl transferase; UD: undetectable

## Discussion

In chronic kidney disease (CKD) stages 4-5 and especially in dialysis patients, progress in HCV infection treatment was slower. Indeed, until a few years ago, SVR rates with the (peg) interferon and ribavirin combinations were around 40% and tolerance was poor, prompting withdrawal of anti-HCV treatment in almost 1/3 of patients [3]. Fortunately, evidence is now accumulating, showing that SVR rates may exceed 95% even in patients on renal replacement therapy [3]. Until recently, there have been few data on the use of DAAs in advanced CKD and particularly in patient on maintenance dialysis. Recent HCV guidelines endorsed the use of initially available DAA regimens only in patients with a glomerular filtration rate (GFR) >30 ml/min. HD patients were precluded from treatment with these drugs. Among the currently approved DAAs, sofosbuvir, a NS5B polymerase inhibitor, is the only DAA which has significant renal elimination. Therefore, there is no sofosbuvir dose recommendation in severe renal insufficiency or in the dialysis setting. There are limited pharmacokinetic data and clinical data reported in few case series regarding the use of sofosbuvir in the HD setting [5-7]. The other currently approved DAAs, simeprevir, ledipasvir, daclatasvir, paritaprevir/ritonavir, ombitasvir, dasabuvir, grazoprevir and elbasvir are not renally eliminated and thus do not need dose adjustment in severe CKD or in HD settings [8]. In our case, given the DAAs available in our setting (sofosbuvir, ledispasvir), the accumulating scientific data on the safety of sofosbuvir in patents on maintenance HD, the multidisciplinary decision and the consent of the patient, he was treated by a sofosbuvir-based regimen. The response was good and no adverse reactions were noticed.

Seventeen patients with ESRD on HD or GFR <30 ml/min received sofosbuvir 400 mg daily and simeprevir 150 mg daily for 12 weeks in a short case series in the United States of America [6]. Treatment was overall well tolerated with no treatment discontinuation reported. Four (24%) patients reported mild adverse events, including: insomnia (n=2), headache (n=1), nausea (n=1) and worsening anemia requiring blood transfusion (n=1). All (n=17) the patients achieved SVR or virological cure (100% SVR). Most common adverse events resembled those of healthier patients with chronic hepatitis C without significant renal impairment [6]. In a case series of 12 French HD patients with chronic HCV infection, patients received sofosbuvir either once daily (n=7) or thrice weekly (n=5) in combination with another agent (ribavirin, simeprevir, daclatasvir or ledipasvir) after dialysis. Ten patients were cirrhotic and 11 of the 12 patients were infected with HCV genotype 1. Despite the high prevalence of cirrhosis, therapy was well tolerated with no serious adverse events. SVR was achieved in 10 of the 12 patients (83%) [9]. No significant accumulation of sofosbuvir was detected on analysis of serial plasma levels in the daily or thrice weekly groups. However, levels of its major metabolite, GS-331007 were 2.5 to 3 times higher in the daily group than in the thrice weekly group when measured pre- and post-HD. Although GS-331007 levels were elevated, no toxicity was linked directly to its accumulation which supports the safety of sofosbuvir in the dialysis population.

Indeed, sofosbuvir is metabolised to the active metabolite GS-461203 which works intracellularly, and subsequently to the inactive metabolite GS-331007, which is the predominant metabolite in plasma [7]. GS-331007 (formerly PSI-6206) is eliminated by the kidneys. Some pharmacokinetic studies showed that this metabolite accumulates in patients on HD with potential toxicity [5,10]. HD extract approximately 15% of sofosbuvir (formerly PSI-7977) and 53% of GS-331007 [10]. In a recent small case series of 2 patients on maintenance HD in Netherland [11], both patients achieved SVR after receiving full-dose sofosbuvir, with good tolerance of the treatment. They did not observe any evidence of hepatobiliary (1.5 fold elevation of aminotransferase or alkaline phosphatase level) or cardiovascular toxicity (occurrence of myocardial infarction/angina/arrhythmia) during treatment. A small study in 10 genotype 1 HCV infected patients with a creatinine clearance <30 ml/min using sofosbuvir 200 mg daily showed low efficacy (SVR: 40%) [5]. Then, lowering the dose seems to reduce the virological response.

Based on these reports sofosbuvir based regimens could be adapted for the treatment of HCV in patients with severe CKD even in the dialysis population [8]. Importantly, our current knowledge of the efficacy and safety of the various doses of sofosbuvir (400 mg daily, 400 mg thrice weekly or 200 mg daily) is based on a few case series with a limited number of carefully selected patients. Data from larger prospective studies are needed in order to determine the optimal dose recommendation of sofosbuvir in advanced CKD and HD patients [8].

## Conclusion

The treatment of HCV infection in patients on maintenance haemodialysis is now possible with most of the new DAAs with great efficiency and tolerance. Unfortunately, these treatments aren´t currently available in Tunisia and other African countries, except a sofosbuvir based regimen. Safe and effective doses of sofosbuvir in patients with an eGFR <30 ml/min have not yet been strongly established. However, there is accumulating evidence on use of sofosbuvir-based regimens in that population. Strong randomized controlled trials and pharmacokinetic/dynamic studies are needed to support future recommendations on that topic of interest.
